The article "Thrombosis in essential thrombocytemia and early/prefibrotic primary myelofibrosis: the role of the WHO histological diagnosis" was published in 2015. Journal: Diagn Pathol.

# Thrombosis in essential thrombocytemia and early/prefibrotic primary myelofibrosis: the role of the WHO histological diagnosis

**DOI:** 10.1186/s13000-015-0269-1

**Published:** 2015-04-16

**Authors:** Serena Rupoli, Gaia Goteri, Paola Picardi, Giorgia Micucci, Lucia Canafoglia, Anna Rita Scortechini, Irene Federici, Federica Giantomassi, Lidia Da Lio, Antonio Zizzi, Elisa Honorati, Pietro Leoni

**Affiliations:** Department of Clinical and Molecular Sciences, Clinic of Hematology, Polytechnic University of Marche Region, Ancona, Italy; Department of Biomedical Sciences and Public Health, Section of Pathologic Anatomy and Histopathology, Polytechnic University of Marche Region, Torrette, Ancona, Italy; Clinical Pathology, United Ancona Hospital, Ancona, Italy

**Keywords:** Essential thrombocytemia, Prefibrotic/early primary myelofibrosis, Vascular events, Histopathology interpretation

## Abstract

**Background:**

Vascular events represent the most frequent complications of thrombocytemias. We aimed to evaluate their risk in the WHO histologic categories of Essential Thrombocytemia (ET) and early Primary Myelofibrosis (PMF).

**Methods:**

From our clinical database of 283 thrombocytemic patients, we selected those with available bone marrow histology performed before any treatment, at or within 1 year from diagnosis, and reclassified the 131 cases as true ET or early PMF, with or without fibrosis, according to the WHO histological criteria. Vaso-occlusive events at diagnosis and in the follow-up were compared in the WHO-groups.

**Results:**

Histologic review reclassified 61 cases as ET and 72 cases as early PMF (26 prefibrotic and 42 with grade 1 or 2 fibrosis). Compared to ET, early PMF showed a significant higher rate of thrombosis both in the past history (22% vs 8%) and at diagnosis (15.2% vs 1.6%), and an increased leukocyte count (8389 vs 7500/mmc). Venous thromboses (mainly atypical) were relatively more common in PMF than in ET. Patients with prefibrotic PMF, although younger, showed a significant higher 15-year risk of developing thrombosis (48% vs 16% in fibrotic PMF and 17% in ET). At multivariate analysis, age and WHO histology were both independent risk-factors for thrombosis during follow-up; patients >60 yr-old or with prefibrotic PMF showed a significantly higher risk at 20 years than patients <60 yr-old with ET or fibrotic PMF (47% vs 4%, p = 0.005).

**Conclusions:**

Our study support the importance of WHO histologic categories in the thrombotic risk stratification of patients with thrombocytemias.

**Virtual slides:**

The virtual slide(s) for this article can be found here: http://www.diagnosticpathology.diagnomx.eu/vs/2020211863144412.

## Background

Essential thrombocythemia (ET) is a clonal stem cell disorder that shares several similarities with other myeloproliferative neoplasms (MPNs), particularly polycythemia vera (PV) and primary myelofibrosis (PMF) [1]. The discrimination between Essential Thrombocythemia (ET) and the early Primary Myelofibrosis (PMF) is especially crucial because it can influence the diagnostic strategies, outcome and complications [2]. The updated WHO classification integrates clinical, molecular and pathological criteria, but the fine morphologic examination of the bone marrow still maintains a central role [3-5]: ET is characterized by a significant increase of enlarged and mature megakaryocytes in a bone marrow with normal cellularity, and normal maturation and quantity of the other series, whereas PMF combines the presence of atypical megakaryocyte proliferation to increased cellularity, increased and left-shifted granulopoiesis, reduced erythropoiesis and/or reticulin and collagen fibrosis. The issue of histologic reproducibility in distinguishing the two diseases has been debated in the literature since 2001 and is still of interest [6-13]. In the present study, we aimed to test the hypothesis that our clinico-pathologic database of patients also contains a mixture of biologically heterogeneous entities with different natural history and clinical outcome in terms of survival and thrombosis: the WHO-defined ET (“true” ET) and early PMF, with different survival and propensity to develop thrombosis during follow-up. By observing a strict adherence to the WHO histologic criteria and blind to clinical data, we reclassified our series as “true” ET and early PMF, and subsequently we subclassified early PMF cases as prefibrotic PMF (grade 0 myelofibrosis) and fibrotic PMF (grade 1 and 2 myelofibrosis). For the significantly higher occurrence of major thrombotic events during follow-up in prefibrotic PMF, we propose a new prognostic model for thrombosis that was based on age and WHO histology.

## Methods

A clinico-pathologic database of patients with complete clinical data consecutively diagnosed as having ET and treated at our institution has been reviewed. This study included 283 patients with ET diagnosed since 1980 and followed up to 2011 at the Clinic of Hematology Polytechnic University of Marche Region, United Hospital of Ancona, Italy. The diagnosis of ET was originally made in accordance with the criteria in use at the time of first observation. In the present study we considered the following parameters: age, sex, platelet count, hemoglobin level, white blood cell count, lactic dehydrogenase (LDH- evaluated in 95 patients), JAK2V617F mutation status (investigated since 2007 in 75 patients), spleen size, history of thrombosis (before and at diagnosis), progression to overt myelofibrosis, conventional risk for thrombosis according to Cervantes [14]. We considered as venous and arterial thrombotic events the following: deep venous thrombosis of the extremities (DVT) or atypical thrombosis (abdominal and cerebral veins), pulmonary embolism (PE), ischemic stroke, cerebral transient ischemic attack (TIA), acute myocardial infarction (AMI) and peripheral arterial thrombosis (PAT).

The histological review was done in cases in whom the bone marrow trephine biopsy was performed before any treatment, at or within 1 year from diagnosis. The histological review was performed on the original slides by a pathologist with 20 year-experience on hematopathology (G.G.) blind to the other clinical and follow-up data. At the time of diagnosis the specimens had been fixed in buffered formalin, decalcified in EDTA and paraffin-embedded. For assessment the histological sections had been stained with hematoxylin and eosin (H&E), Giemsa, periodic acid Schiff reagent (PAS), Prussian Blue and Gomori’s silver impregnation. Of each specimen, the following parameters were considered according to Thiele and Kvasnicka [6]: the overall bone marrow cellularity compared to the age-matched control [15], the amount of granulopoiesis, erythropoiesis and megakaryocytopoiesis (scored as 0 for normal or reduced, 1 for slight increase, 2 for moderate increase, 3 for marked increase); left-shifted maturation of erythroid and myeloid series (absent or present); clusters of megakaryocytes (absent, loose or dense); giant hyperlobulated or bulbous MGKs (absent, rare or frequent); reticulin fibrosis according to a 4-graded system [15]: 0 for scattered linear reticulin with no intersections (cross-overs); 1 for a loose network of reticulin with many intersections, especially in perivascular areas; 2 for diffuse and dense increase in reticulin with extensive intersections, occasionally with only focal bundles of collagen and/or focal osteosclerosis; 3 for diffuse and dense increase in reticulin with extensive intersections with coarse bundles of collagen, often associated with significant osteosclerosis. In all cases immunostainings for myeloid, erythroid and megacariocytic markers were also performed to better evaluate these parameters. When necessary, histochemical and immunohistochemical stainings were repeated. All cases were reclassified as “true” ET and early PMF in their turn divided into prefibrotic PMF (grade 0 myelofibrosis) and fibrotic PMF (grade 1 and 2 myelofibrosis) according to 2008 WHO morphologic criteria [4,5].

### Statistical analysis

Statistical analysis was performed with SPSS software for Windows (Statistical Product and Service Solutions, version 14.0, SSPS Inc, Chicago, IL, USA). The clinical and histologic parameters were compared in the histological categories. Quantitative variables were expressed as mean values and standard deviation (SD) for normally distributed data. These data were compared using the Mann–Whitney test. Differences between the qualitative variables were evaluated using the chi-square test. P < 0.05 was considered statistically significant. The Kaplan-Meier product-limit method was used to estimate univariate survival curves, and the log-rank test was selected to compare the survival curves. Cox proportional hazards regression was used to perform multivariate survival analyses. Risk of thrombosis was reported as by cumulative incidences calculated at 5, 10, 15 and 20 years from the date of diagnosis. Overall survival (OS) analysis was considered from the date of diagnosis to date of death or last contact. Event-free survival curves were calculated from the date of diagnosis to date of leukemic transformation or progression into overt myelofibrosis, or last contact/date of death.

## Results

A total of 142 cases were considered for the present study. In 61 (43%) the histology was consistent with a diagnosis of ET (Figure 1A), 72 (51%) were revised to early PMF (Figure 1B), and 9 cases (6%) were excluded from the analysis as they did not exhibit discriminating features between the two categories and considered as unclassifiable MPNs. In PMF cases, 46 cases were fibrotic (grade 1 and 2) and 26 were prefibrotic (grade 0). All early PMF with the exception of four cases, lacked the minor clinical criteria for PMF stated in the WHO classification (leukoerythroblastosis, increase in serum LDH level, anemia, and splenomegaly). Median follow-up from time of diagnosis was 117 months (95% C.I., 103–144) for ET and 85 months (95% C.I., 85–119) for early PMF (p not significant). Table 1 provides a comparison of the clinical, laboratory and histological parameters for patients with ET and those with early PMF. Significant differences were seen for mean leukocyte count (higher in early PMF than ET: 8389 vs 7500; p = 0.001), history of thrombosis (more frequently in early PMF than ET: 22% vs 8%; p = 0.032) and thrombosis at the onset of disease (more frequently in early PMF than ET: 15.25% vs 1.6% respectively; p = 0.006). Mean semiquantitative score referring to granulopoiesis was significantly different (greater in early PMF than ET: 1.02 vs 0.15; p = 0.001); moreover we found a significant correlation between granulopoiesis scores and thrombosis at the onset of disease (Mann–Whitney test, 0.60 without thrombosis vs 1.10 with thrombosis, p < 0.05). JAK2V617F mutational frequencies were also different between the two groups although without statistical significance (greater in early PMF than ET: 54% vs 33%; p = 0.06). On the contrary age, sex distribution, anemia, LDH serum values, palpable spleen and thrombotic complications during follow-up, were similar between the two groups. Table 2 shows that venous thrombosis (mainly atypical) were relatively common in early PMF, as opposed to ET. In this regard, it must be pointed out that almost all of the abdominal thrombosis (in total 5 cases out of six) were JAK2V617F positive. Table 3 describes the epidemiological and clinical characteristics of the two PMF subgroups. Neither hematologic data nor frequency of previous thrombosis was significantly different between fibrotic versus prefibrotic PMF patients with the exception of age, given that patients with prefibrotic PMF were significantly younger (43 years and 61 years; p < 0.019).

**Figure 1:** H&E of bone marrow in ET **(A)** and in grade 0 Prefibrotic PMF **(B)**. Original magnification x20. In cases considered ET, the cellularity appeared not increased, the megakaryocytes were mainly giant with stag-horn like nuclei and showed low tendency to aggregate. In cases considered PMF, the cellularity was increased mainly for expansion of granulopoiesis; the megakaryocytes were aggregated and showed frequently hypolobulated nuclei.

**Table 1:** **Clinico-pathological parameters for patients with ET and early/prefibrotic PMF**

	**True ET**	**PMF**	***p value***
M/F	27/34	26/46	n.s.
Median age (years)	58.0 (23–84)	55.5 (20–87)	n.s.
Mean WBC (10^9^/l)	7.5	8.4	*p = 0.001*
Mean Hb (g/dl)	14.1	14.3	n.s.
Mean PLT (10^9^/l)	751	798	n.s.
Increased LDH (%)	17/45 (37.7%)	18/50 (36.0%)	n.s.
Splenomegaly (%)	12 (19%)	18 (25%)	n.s.
Mean semiquantitative score for granulopoiesis	0.15	1.02	*p = 0.001*
JAK2V617F-positive (%)	11 (33%)	23 (54%)	n.s.
History of thrombosis (%)	5 (8%)	16 (22%)	*p = 0.032*
Thrombosis at diagnosis (%)	1 (1.6%)	11 (15.2%)	*p = 0.006*
Thrombotic events during follow up (%)	7 (11.4%)	11 (15.2%)	n.s.
Progression to overt MF (%)	1 (1.6%)	3 (4.1%)	n.s.
Dead/alive	2/59	8/64	n.s.
Conventional Risk (Low/High)	35/26	30/42	n.s.
Cytoreductive therapy (%)	51 (83%)	64 (88%)	n.s.

**Table 2:** **Main thrombotic events at diagnosis and during follow up in ET and PMF**

**Thrombotic events at diagnosis**							
	**AMI**	**Stroke, TIA**	**Retinal occlusion, PAT**	**DVT**	**PE**	**Splanchnic vein thrombosis**	**Cerebral thrombosis**
ET	1						
PMF	2	1	1	3		3	1
**Thrombotic events during follow-up**							
ET	2	4		1			
PMF	2	2	2	1	1	3	

Note: AMI = acute myocardial infarction; TIA = transient ischemic attack; PAT = peripheral arterial thrombosis; DVT = deep-vein thrombosis; PE = pulmonary embolism.

**Table 3:** **Clinical characteristics in the two subgroups of prefibrotic and fibrotic PMF**

	**Prefibrotic PMF**	**Fibrotic PMF**	***p value***
Sex	M:F = 11/15	M:F = 15/31	n.s.
Median age at diagnosis (years)	43 (20–87)	61 (27–83)	*p = 0.019*
WBC at diagnosis (10^9^/l)	9100	8745	n.s.
Hb at diagnosis (g/dl)	14.6	14.3	n.s.
PLT at diagnosis (10^9^/l)	825000	797500	n.s.
Increased LDH	6/19 (31.6%)	19/31 (61.3%)	n.s.
Splenomegaly (%)	6 (23%)	12 (26%)	n.s.
JAK2V617-positive (%)	9 (50%)	14 (58%)	n.s.
History of thrombosis (%)	6 (23%)	10 (22%)	n.s.
Thrombosis at diagnosis (%)	4 (15%)	7 (15%)	n.s.
Thrombotic events during follow-up (%)	6 (23%)	5 (10%)	n.s.
Progression to overt MF (%)	0 (0%)	3 (6.5%)	n.s.
Dead/Alive	2/24	6/40	n.s.
Conventional Risk (Low/High)	13/13	17/29	n.s.
Cytoreductive therapy (%)	24 (92%)	40 (86%)	n.s.

During the follow-up period, 2/61 patients with ET and 8/72 with early PMF had died (p not significant). Cytoreductive therapy was applied in 51 patients (83%) with ET and in 64 (88%) with early PMF (p not significant) (Table 1). In total overt fibrotic transformations were documented in one patients (1%) and 3 patients (4%), respectively, with ET and with early PMF (p not significant). At 15 years, overall survival was significantly better in ET than in early PMF, respectively 96% vs 76% (p = 0.027). Multivariate analysis showed that only age over 60 years and histology (early PMF) were significant risk factors for reduced overall survival (p < 0.05).

Progression to overt myelofibrosis and leukemia (PFS) and death rates were similar between the 2 subgroups of PMF and ET patients, whereas ET patients showed a significantly superior OS only than fibrotic PMF (Figure 2). During follow-up, patients with prefibrotic PMF, although younger, showed a significant higher risk of developing thrombosis: the 15-year risk of thrombosis was 48% in prefibrotic PMF, 16% in fibrotic PMF (grade 1, 2) and 17% in ET (prefibrotic PMF vs fibrotic PMF p = 0.049; prefibrotic PMF vs ET p = 0.032; Figure 3). Multivariate analysis confirmed that prefibrotic PMF is an independent risk factor for cumulative thrombotic events and identified age older than 60 years as an additional risk factor for thrombosis (p < 0.05). According to our data, we propose a new risk score: patients older than 60 or those with prefibrotic PMF are high risk patients, whereas those younger and with ET and fibrotic PMF should be considered at low risk. By applying the model to our series at diagnosis, the development of future vascular events is 34% and 7% for high and low risk at 15 years (p = 0.005) and 47% and 7% for high and low risk at 20 years (p = 0.005; Figure 4).

**Figure 2:** Overall survival (OS) of patients with ET, prefibrotic PMF and fibrotic PMF. Significant differences were found only between ET and fibrotic PMF patients (p = 0.027).

**Figure 3:** Risk of thrombosis during follow-up: the 15-year risk of thrombosis was 48% in prefibrotic PMF, 16% in fibrotic PMF (grade 1, 2) and 17% in ET. Differences were significant between prefibrotic PMF vs fibrotic PMF (p = 0.049) and between prefibrotic PMF vs ET (p = 0.032).

**Figure 4:** Patients older than 60 or with prefibrotic PMF are high-risk patients, whereas those younger and with ET and fibrotic PMF should be considered at low risk. The resulting risk categories (high or low-risk) better predicted future vascular events than conventional risk factors (34% and 7% respectively for high and low risk at 15 years; p = 0.005).

## Discussion

Many literature data, mainly arising from the Cologne Group, showed that approximately 40% to 50% of patients with clinical “ET” have an initial stage of PMF presenting with thrombocytosis and characterized by prominent granulocytic and megakaryocytic proliferation and significant anomalies of megakaryocytes [10]. In our study the review of initial bone marrow specimens, confirmed ET diagnosis in only 43% and changed to early PMF in 50% and is in line with these data. The relevance of a sharp distinction of ET and early PMF is stressed by clinical results of Barbui et al. in an international-based data collection of 1104 patients with a clinical phenotype of ET [2]: WHO-defined ET patients showed a lower risk of overt myelofibrosis, AML evolution, and, finally, a better survival compared with PMF. The discussion on the reproducibility of the WHO-subjective morphological criteria is still ongoing, as for many authors these criteria are not simple to apply [8,9,11], whereas for others an agreement among pathologists can be achieved in 88% to 93% of cases [10,12,13]. In our study the issue of the inter-observer histologic reproducibility was beyond our aims, although it may be considered a potential bias. In reality, as the original diagnoses were made by a group of general pathologists with different degree of expertise in the field and were reviewed in approximately 60% of cases by a single expert hemopathologist from the same department, we believe that it offers the perspective of the diagnostic work in the daily-practice by general practitioners and referral pathologists, pointing out the importance of careful clinico-pathological correlation in patient with MPNs [16].

In our series, at diagnosis, early PMF patients showed greater leukocyte count, history of thrombosis and thrombosis at the onset of disease, than ET patients. Statistical analysis of morphological features (semiquantitative scoring system) and clinical data showed a significant correlation between medullary leukocytosis and thrombosis. Multivariate analysis undoubtedly states that histology (early/prefibrotic PMF) is a predictor of reduced survival as well as age over 60 years. It is well known that Thiele and co-workers [10] first stated that BM fibrosis is not an intrinsic and necessary marker of PMF, and proposed a new category of patients with dual megakaryocytic and granulocytic myeloproliferation associated with characteristic megakaryocyte dysplasia and absence of relevant reticulin fibrosis in BM. This variant with BM fibrosis grade 0 was called prefibrotic myelofibrosis whereas the variant with the BM morphological features of early PMF but having at least grade 1 fibrosis was categorized into the fibrotic type category of PMF. In the present study progression (to overt myelofibrosis and leukemia) and death rates were similar between the fibrotic and prefibrotic early PMF, while WHO-ET patients showed a significantly superior OS than fibrotic PMF. Furthermore, statistical analysis allowed us to recognize that prefibrotic PMF patients, although younger, presented with a higher probability of thrombotic events (48%) compared with WHO-ET (16%) or fibrotic PMF patients (17%). Some characteristics of our prefibrotic PMF show striking similiarities with those that were well-outlined in the series of Barosi [17,18]. The mobilization of endothelial progenitors (ECFCs) cells is consistently higher in patients who received a diagnosis of prefibrotic myelofibrosis, thus giving rise to the hypothesis that endothelial progenitor cell-mediated neoangiogenesis, could intervene in determining the distinctive phenotypic profile of prefibrotic PMF [19]. As for thrombotic risk, until now, the incidence of thrombosis in prefibrotic PMF have been rarely assessed. Barbui et al. [20] showed that the rate of major cardiovascular events in PMF was comparable with that reported in ET, and it was increased in aged patients and those with JAK2V617F mutation and leukocytosis. Unfortunately in that study, the so-called “prefibrotic” form of PMF was not considered. In the same year, Brousseau et al. [9] applied WHO criteria to bone marrow specimens of patients previously diagnosed as having ET and observed no clinical (including thrombosis) or biologically differences between “true ET”, prefibrotic and fibrotic PMF. The clinical course of 264 patients with early/prefibrotic PMF was subsequently studied by Buxhofer-Ausch and co-warkers [21]; the authors suggested the importance of early/prefibrotic PMF as a distinct sub-entity of MPNs and indicated that leukocytosis at diagnosis was the preminent risk of total and arterial thrombosis in particular. Initial bone marrow reticulin fibrosis also exerts an impact on clinical outcome in polycythemia vera [22]. Barbui found a significantly higher occurrence of major thrombotic events during follow-up, in PV patients without reticulin fibrosis; on the contrary PV patients with increases in reticulin fibrosis displayed a higher prevalence of palpable splenomegaly and were more prone to develop overt myelofibrosis. The authors speculated that the variant without reticulin fibrosis might be characterized by a different biology or that the higher rate of thrombotic events might be related to a longer disease duration [22]. The major consequence of these findings is that the prefibrotic forms of PV and PMF could be considered acquired thrombophilic conditions, potentially requiring a new way of therapeutic intervention. Current thrombosis risk factors in ET are age and previous vascular events [23-26] and mutational status for JAK2, MPL, and Calreticulin [27]. Our study provides evidence that a morphologic discrimination of prefibrotic PMF from true ET has a significant impact on the risk of thrombosis. At multivariate analysis, among the potential predictors, only age and histopathology remained independent risk factors for thrombosis during follow-up. Patients older than 60 or with prefibrotic PMF are high-risk patients whereas those younger and with fibrotic PMF or true ET should be considered low-risk. Whether our new risk classification may optimize the management of patients presenting clinically with “ET” needs to be validated in association with mutational analysis. If prefibrotic PMF is strongly affected by thrombosis, its recognition might favor an early intervention at the time of diagnosis, to reduce MPN clone-derived prothrombotic features. Probably it is time to better understand the characteristics of prefibrotic PMF, change our “wait and watch strategy” [28] and start an upfront therapy (e.g. IFN-α [29] as monotherapy or in addition to JAK_2_-inhibitors) combined with the treatment of all modifiable factors that increase the vascular risk [30]. Moreover, the antithrombotic effectiveness of aspirin, demonstrated in PV and to a lesser extent in ET [31,32], might be tested in prefibrotic PMF after a careful evaluation of the individual hemorrhagic risk.

## Conclusions

Our study provides further evidence that morphologic features of the bone marrow favoring the diagnosis of prefibrotic PMF or true ET, have a significant impact on the risk of thrombosis. Bone marrow histologic examination should maintain a central role in the diagnostic and therapeutic approach of patients with thrombocytemias.
